The article "Effect of pH on the Electrochemical Behavior of Hydrogen Peroxide in the Presence of Pseudomonas aeruginosa" was published in 2021. Journal: Front Bioeng Biotechnol.

# Effect of pH on the Electrochemical Behavior of Hydrogen Peroxide in the Presence of *Pseudomonas aeruginosa*

**DOI:** 10.3389/fbioe.2021.749057

**Published:** 2021-12-06

**Authors:** Javier Espinoza-Vergara, Paulo Molina, Mariana Walter, Miguel Gulppi, Nelson Vejar, Francisco Melo, Marcela Urzua, Hugo Muñoz, José H. Zagal, Xiaorong Zhou, Manuel I. Azocar, Maritza A. Paez

**Affiliations:** ^1^ Departamento de Química de Los Materiales, Facultad de Química y Biología, Universidad de Santiago de Chile, Santiago, Chile; ^2^ Corrosion and Protection Center, Department of Materials, University of Manchester, Manchester, England, United Kingdom; ^3^ Chilean Air Force, Aerospace Sciences Research and Development Centre (CIDCA), San Bernardo, Santiago, Chile; ^4^ Departamento de Física, Facultad de Ciencias, Universidad de Santiago de Santiago de Chile, Avenida Ecuador, Santiago, Chile; ^5^ Facultad de Ciencias, Universidad de Chile, Santiago, Chile

**Keywords:** *pseudomonas aeruginosa*, catalase, hydrogen peroxide, cobalt phthalocyanines, oxygen reduction

## Abstract

The influence of pH on the electrochemical behavior of hydrogen peroxide in the presence of *Pseudomonas aeruginosa* was investigated using electrochemical techniques. Cyclic and square wave voltammetry were used to monitor the enzymatic activity. A modified cobalt phthalocyanine (CoPc) carbon electrode (OPG), a known catalyst for reducing O_2_ to H_2_O_2_, was used to detect species resulting from the enzyme activity. The electrolyte was a sterilized aqueous medium containing Mueller-Hinton (MH) broth. The open-circuit potential (OCP) of the *Pseudomonas aeruginosa* culture in MH decreased rapidly with time, reaching a stable state after 4 h. Peculiarities in the E / I response were observed in voltammograms conducted in less than 4 h of exposure to the culture medium. Such particular E/I responses are due to the catalase’s enzymatic action related to the conversion of hydrogen peroxide to oxygen, confirming the authors’ previous findings related to the behavior of other catalase-positive microorganisms. The enzymatic activity exhibits maximum activity at pH 7.5, assessed by the potential at which oxygen is reduced to hydrogen peroxide. At higher or lower pHs, the oxygen reduction reaction (ORR) occurs at higher overpotentials, i.e., at more negative potentials. In addition, and to assess the influence of bacterial adhesion on the electrochemical behavior, measurements of the bacterial-substrate metal interaction were performed at different pH using atomic force microscopy.

## Introduction

In general, the degradation of materials involves chemical and/or electrochemical processes at the material-environment interface (Nash et al., 2018). The presence of biological fluids, liquids or gases, and microorganisms, which colonize the surface of metallic structures, also affect their degradative behavior. (Hamilton, 1998; Busalmen et al., 2002; Wang et al., 2006; Rosales and Iannuzzi, 2008; Little and Lee, 2014; Gilbert, 2020). The different metal-environment combinations resulting from considering other metals and distinct environments (aqueous liquids, organic liquids, humid gaseous atmospheres, biological fluids, etc.) give rise to highly complex metal-environment interfaces.

In particular, when microorganisms intervene in the degradation of materials, the complexity is even more significant because the production of metabolites and species that result from the evolution and survival mechanism of the microorganism intervenes in the degradation process. Hydrogen peroxide (H_2_O_2_) is continuously formed by the autoxidation of redox enzymes in aerobic cells, and it also enters from the environment, where it can be generated both by chemical processes and by the deliberate actions of competing organisms. Because H_2_O_2_ is acutely toxic, bacteria elaborate scavenging enzymes to keep its intracellular concentration at nanomolar levels (Chelikani et al., 2004; Mishra and Imlay, 2012).

Mutants that lack such enzymes grow poorly, suffer from high mutagenesis rates, or even die (Chelikani et al., 2004). Further, the catalytic effect promoted by the mutated microorganisms (*Escherichia coli*), deficient in catalase, is markedly inhibited (Baeza et al., 2013).

In order to understand how bacteria cope with oxidative stress, it is essential to identify the key enzymes involved in hydrogen peroxide (H_2_O_2_) degradation. Catalases and nicotinamide adenine dinucleotide peroxidase (NADH peroxidase) are primary scavengers in many bacteria, and their activities have been unambiguously demonstrated through phenotypic analysis and through direct measurements of H_2_O_2_ clearance *in vivo* (Sepunaru et al., 2016; Erttmann and Gekara, 2019).

The oxidative stress hypothesis postulated in the last 30 years establishes that oxygen toxicity is mainly mediated by partially reduced oxygen species, more reactive than molecular oxygen itself. Both calculations and experiments indicate that microbes have acquired sufficient defensive measures to avoid overt poisoning by endogenous reactive oxygen species (ROS) (Erttmann and Gekara, 2019). Any elevation in the intracellular levels of these oxidants, particularly superoxide (O_2_^−^) and hydrogen peroxide (H_2_O_2_), produces enough enzyme damage to stop the growth and enough Deoxyribonucleic acid (DNA) damage from accelerating mutagenesis. A survival mechanism is then triggered that involves the release of enzymes.

The enzymes generated transform hydrogen peroxide into oxygen and water *via* dismutation. However, the results do not always provide a consensus. The purpose of this work is to demonstrate through a simple electrochemical experiment the relationship between partially reduced oxygen species, particularly hydrogen peroxide, and the enzymatic defense mechanism of a catalase positive bacteria, such as *P. aeruginosa*.

For the evaluations of the enzymatic activity of catalase-positive microorganisms, we have used some electrochemical techniques, such as cyclic voltammetry (CV) and differential pulse voltammetry (DPV), using as sensor surfaces of pyrolytic graphite electrode modified with CoPc. The electrochemical behaviors of the “metallic surface-electrolyte” interfaces were studied in the absence and presence of microorganisms, mainly *Escherichia coli* and *Staphylococcus aureus*. Such investigations show that the catalase enzyme present in microorganisms is activated almost instantaneously when hydrogen peroxide is deliberately added to the electrolyte. (Gulppi et al., 2019). Further, in the previous experimental research, the pH markedly influenced the electrochemical response of the studied systems. Regarding the mentioned pH influence, the enzymatic mechanism is studied in this work but examines the pH effect on the electrochemical response.

The pH effect in charge transfer reactions that involve the reduction of oxygen or partially reduced oxygen species (peroxides or superoxides) is known and expected, given the participation of H^+^ ions and/or OH^−^ ions in the half-reactions of oxide-reduction. In the particular case of the pH effect on the activity of enzymes, they are also sensitive to pH. The change in pH in its environment could change the shape of the active site of an enzyme and contribute to the folding of the enzyme molecule (Chelikani et al., 2004; Mishra and Imlay, 2012; Erttmann and Gekara, 2019). Changes in the active site form may decrease its ability to bind to the substrate and cancel its function as an enzyme (catalase in this case). Each enzyme has an optimal pH value where it reaches its maximum activity, called the optimum pH. If the pH is lower or higher than the optimum pH, the enzyme activity decreases until it is inactivated. Several works have been carried out to study the optimum pH of the activity of a wide range of enzymes (Shahani, 1966; Frankenberger and Johanson, 1982; Silvestre et al., 2012; Bhalla et al., 2015). Nevertheless, many enzymes, especially those from mammalian sources, possess a pH optimum near the physiological pH of 7.5 (Bisswanger, 2014).

At extremely high pH levels, the charge of the enzyme is altered, and consequently, its solubility and general shape. Regarding catalase, it is hypothesized that the optimal pH range for the catalytic operation of the enzyme is between pH 6 and 8 (Chance, 1952).

Various methods have been proposed to measure the growth of bacteria, such as measurement of molecular oxygen consumption (Zlatev et al., 2013; Gulppi et al., 2019), peroxide production (McLeod et al., 1922; Ferenci, 1999; Reichart et al., 2007), and open circuit potential measurements (Zlatev et al., 2013). The investigations carried out in our previous work (Baeza et al., 2013; Gulppi et al., 2019) have shown that it is possible to interrelate the information provided by these techniques with interfacial processes associated with material degradation assisted by catalase activity in the decomposition of H_2_O_2_ to O_2._ Then, following our previous work, and expanding the study to another positive catalase microorganism, *P. aeruginosa*, in this work, cyclic voltammetry (CV) and square wave voltammetry (SWV) is employed to study the influence of pH on the enzyme activity. Like other catalase-positive bacteria, *P. aeruginosa* is expected to spontaneously produce catalase in response to the oxidative stress promoted by hydrogen peroxide (Figure 1), and in this way, to keep its intracellular concentration at a nanomolar level. Further, to make catalase activity even more noticeable and detect O_2_ as a decomposition product, an excess of H_2_O_2_ was deliberately added. We used a modified carbon electrode (OPG) with CoPc as a sensor to monitor the electroreduction of oxygen. CoPc promotes the reduction of O_2_ to peroxide only (Zagal et al., 1992; Baeza et al., 2013; Zagal et al., 2014; Zagal and Koper, 2016; Gulppi et al., 2019).

**FIGURE 1:** Open circuit potentials obtained in the absence (Control/black line) and presence (red line) of *P. aeruginosa* in 100 ml of Mueller-Hinton broth at pH 7 in a solution previously saturated with O_2_.

Regarding the influence of pH and considering that enzymatic activities could also result from the effect of pH on the adherence of the microorganism, an atomic force microscopy study was carried out to determine the bacterial adherence forces at different pH’s. Such studies were carried out on aluminum alloy surfaces considering 1) the lower roughness of these surfaces compared to the (OPG) electrode surfaces and 2) the evidence of biodegradation of these materials in the presence of *P. aeruginosa*.

## Experimental Procedure

### Preparation of Culture Broth

The bacterial culture was prepared in a Mueller-Hinton (MH) broth (Merck). MH medium containing: beef extract (8.8% w/w), casein hydrolysate (77% w/w), starch (6.6% w/w), and agar (7.5%w/w).

21 g of the MH medium was dissolved in 1 L of distilled water; the resulting mixture was sterilized in an autoclave for 15 min at 121°C.

Prior to electrochemical experiments, 100 ml of the sterilized mixture, and aliquot of 1 ml of the bacterial culture of *P. aeruginosa* (ATCC 15442) was added, at 37°C with shaking for 24 h.

### Electrochemical Measurements

The potentiodynamic measurements were carried out with an Autolab PGSTAT30 potentiostat/galvanostat. All materials, both liquid and solid, were sterilized before use. The electrolyte was autoclaved at 120°C for 20 min, while the electrodes and the electrochemical The cells were washed with ethanol (70% v/v) three times and exposed to ultraviolet light (254 nm, 20 W, Hg vapor lamp) for 15 min. A conventional three electrode electrochemical cell configuration was used for cyclic and square wave voltammetry measurements. A platinum counter electrode (platinum wire coil of 8 cm^2^ area) was used, Ag/AgCl, (reference electrode 3.5 M) was the reference, and the working electrode was pyrolytic graphite with an area of 0.2 cm^2^. The working electrode was modified with CoPc, which was adsorbed on the surface to sense hydrogen peroxide. The adsorption process was carried out at room temperature by placing an aliquot of 10^–4^ M CoPc solution in dimethylformamide in contact with the electrode’s surface for 5 min. After surface modification, the working electrode was washed with ethanol to remove any excess of CoPc. Electrochemical measurements of OCP in sterilized (without bacteria) and inoculated media (previously sterilized) with bacteria *P. aeruginosa*.

After placing the corresponding electrodes on the sterilized media without bacteria and inoculated with the bacterium *P. aeruginosa*, the electrochemical cell was hermetically sealed during the whole experiment.

Bacterial numbers were determined by spectrophotometric measurements of absorbance at 600 nm and calculated as colony-forming units per milliliter (CFU/ml) by McFarland Method (0.5 OD / 5 × 10^5^ CFU/mL) (Baeza et al., 2013; Gulppi et al., 2019). The inoculated medium was used in exponential phase (OD 0.5) after 5 h of incubation at 37°C. All electrochemical measurements were repeated five times, and the measured values and plotted correspond to the averages.

### Bacterial Adhesion Assessment

Bacteria were first imaged on an aluminum surface. Atomic force microscopy (AFM) images of cells deposited on AA 2024 and AA 6063 aluminum alloys were obtained in the air using the Nanoscope III instrument (Digital Instruments) in the tapping mode, using J scanner. Olympus AC240TS silicon nitride cantilever, with a resonance frequency of 70–100 kHz, a radius of curvature of 20 nm, and stiffness of 5 N/m, was used at a scanning speed of 1 Hz. The cells were cultured in a Muller-Hinton broth in Falcon tubes containing alloy sheets previously washed with phosphate-buffered saline (PBS) at 37°C for 24 h. After the exposure, the aluminum alloy surfaces exhibited relatively well-developed biofilms. Before imaging, samples were rinsed with copious milli-Q water and air-dried in a clean environment maintained at 30 % relative humidity.

Silicon nitride cantilevers with a sphere of SiO_2_ of 5 nm in diameter at one end (purchased from Novoscan PTGS) were immersed for 2 min in drops of 1% (v/v) Polyethylenimine solution (PEI). This procedure was performed to evaluate cell adhesion. After removing excess of the solution, the probes were dried with N_2_ gas and stored at 4°C in a darkened non-frost- free refrigerator until use. For immobilizing bacteria on the colloidal probe, harvested as described above, pelleted cells were manually transferred to the PEI coated microsphere, using a micromanipulator (Narishige MHW-3), under a Nikon inverted microscope. A Nanoscope III AFM, operated in contact mode, was used to measure the adhesion force between the colloidal sphere previously coated with the bacteria and the two aluminum alloy surfaces coated with the bacteria. Scheme 1 schematizes the colloidal probe configuration.

**SCHEME 1:** Features of the force extension curve used for the estimation of adhesion work, W_adh_. Inset: Sketch of the colloidal probe inseminated with bacteria, showing the principle employed for the testing of the bacteria-alloy adhesion.

Adhesion measurements were carried out preparing phosphate buffer solutions at different pH (5,5 to 7,5) and then placing the bacterial inoculum. The tensile force measurement was carried out by activating AFM with a scan frequency of 0.3 Hz and zero scan size. The ramp’s size was approximately 300 nm, and the loading force was applied by setting the maximum deflection value (maximum force on bacteria was approximately 10 nN). Care was taken to minimize lateral force and keep the vertical compression force small on approach to limit the cell probe’s damage. Several force curves were automatically acquired at different locations on the alloy surface by moving the cantilever laterally by an incremental step distance of 50 nm. In this way, sufficient statistical data were obtained.

Various sectors of the sample were measured to ensure representative statistics on the macroscopic surface. From the cantilever deflection curves, the maximum tensile force was obtained by multiplying the maximum cantilever deflection by the cantilever stiffness. The thermal fluctuation method was used to obtain cantilever stiffness.

The work of adhesion, W_adh_, is evaluated as the total energy necessary to completely separate the bacterium body from the aluminum surface. Schema 1 schematizes how the work of adhesion is evaluated through the measurement of the force of adhesion, F, which is integrated over the distance, z, between the cell and the alloy surface. In the schema 1, the interval of distances [L_0_, L_adh_] accounts for the whole range of interaction, for which the cell is under tension, and F_adh_ is the maximum force of adhesion. Thus, in schema 1, the hatched zone represents the work of adhesion.

It should be noticed that this definition of work of adhesion is suitable in the present study since it considers that the main source of adhesion comes from the pilus stretching and its unzipping [ (Knight et al., 1998; Pratt and Kolter, 1998; Cavalcanti-Adam et al., 2006)]. In addition, it is worth mentioning that our definition differs from that provided by the theory of Johnson, Kendall, and Robert (Butt et al., 2005), which applies when the cell body deforms elastically due to the force of adhesion.

## Results and Discussion

### Open Circuit Potential

Figure 1 shows the open circuit potential (OCP)-time response in Mueller-Hinton (MH) culture broth in the absence and presence of *Pseudomonas aeruginosa* in the presence of a solution previously saturated with oxygen, purging the solution for 2 hours.

The OCP measurement in the microorganism’s presence started immediately after adding a 1 ml of the culture inoculum containing *P. aeruginosa* to 100 ml MH culture broth. The OCP decreases markedly in the first 2 h, because of the gradual decrease of oxygen concentration in the electrolyte. *P. aeruginosa* has five terminal oxidases for aerobic respiration (Comolli and Donohue, 2002; Comolli and Donohue, 2004). These terminal oxidases are expected to have their specific affinity for oxygen, since *P. aeruginosa* uses oxygen as an electron receptor in its metabolic processes. (Arai, 2011).

Furthermore, from Figure 1, it can be seen that after approximately 2 h, the potential value increases again sharply to a maximum of -150 mV, exhibiting OCP peculiar behavior (see the graphic inset in Figure 1) that is discussed below. After approximately 240 min, the OCP remained relatively stable during the rest of the measurement. The bacterial culture solution reached pseudo-thermodynamic equilibrium with the environment (open system) at a potential of approximately -173 mV (vs. Ag/Ag/Cl 3.5 M).

Figure 2 shows the OCP-time response in MH medium inoculated with *P. aeruginosa* at different pHs. At pH 6.5, the OCP-time response is similar to that at pH 7.0 shown in Figure 1; the potential falls sharply at the beginning, then increases steeply to a maximum to form a peak. This peculiar behavior, as previously mentioned, is associated with converting hydrogen peroxide to oxygen and is not observed at the other pHs, suggesting that catalase’s action is favored at neutral pH, in agreement with previous work (Gulppi et al., 2019). The interrelation between the generation of hydrogen peroxide by bacteria and the generation of oxygen resulting from catalase action has been demonstrated for two positive catalase microorganisms, *Escherichia coli* and *Staphylococcus aureus* (Gulppi et al., 2019). The experiment consisted of simultaneously sensing the OCP and the medium’s oxygen concentration, using a Clark probe, and following the procedure described by Zlayev et al. (Zlatev et al., 2013). Oxygen concentration and OCP in the culture media are closely associated with microbial culture growth (Zlatev et al., 2013; Gulppi et al., 2019), independent of the bacterial type strain.

**FIGURE 2:** Open circuit potentials obtained in 100 ml of Mueller-Hinton broth with 1 ml of bacterial culture at different pHs in a previously saturated with O_2_.

### Measuring the Enzymatic Activity of Catalase

Previous research (Baeza et al., 2013; Gulppi et al., 2019) by the authors has shown that enzyme activity can be determined in aqueous solutions in the presence of microorganisms, mainly bacteria. In these studies, the E / I response has been measured in voltammetric scans, using a working electrode made of pyrolytic graphite modified with surface-confined CoPc. During cathodic polarization, CoPc catalyzes the reduction of oxygen in two consecutive steps of 2 electrons each, according to the following reactions (written for acid solution):

$$O_{2}+2H^{+}+2e^{-}\to H_{2}O_{2}$$ (1)

$$H_{2}O_{2}+2H^{+}+2e^{-}\to 2H_{2}O$$ (2)

On the other hand, monofunctional catalases that contain a heme group (Fita and Rossmann, 1985) exhibit a common two-step mechanism for the degradation of H_2_O_2_. In a first step, a hydrogen peroxide molecule oxidizes heme (in catalases that contain heme) to an oxyferryl (involving the oxidation of Fe(III) to Fe(IV)). An oxidation equivalent of iron is removed, and another of the porphyrin ring, to generate the cationic porphyrin radical: (Eq. 3).

$$\mathrm{Enz}\left(\mathrm{Por}-Fe^{\mathrm{III}}\right)+H_{2}O_{2}\to \mathrm{Compound}\;I\left(\mathrm{Po}r^{+}-Fe^{\mathrm{IV}}=O\right)+H_{2}O$$ (3)

A second hydrogen peroxide molecule is utilized as a reductant of compound (I) to regenerate the resting-state enzyme, water, and oxygen (Eq. 4).

$$\mathrm{Compound}\;I\left(\mathrm{Po}r^{+}\mathrm{-F}e^{\mathrm{IV}}=O\right)+H_{2}O_{2}\to \mathrm{Enz}\left(\mathrm{Por}-Fe^{\mathrm{III}}\right)+H_{2}O+O_{2}$$ (4)

Despite this common reaction mechanism, enzymatic activities are very different among the various monofunctional catalase genes present in the bacterium *P. aeruginosa*. These are nominally differentiated as katA, katB, and katE. The main catalase katA is the most inducible against the damaging effect of hydrogen peroxide and is present in *P. aeruginosa* (Ochsner et al., 2000; Klotz and Loewen, 2003). We cannot refer to that type of catalase that releases the microorganism, but we can study the enzymatic activity associated with the enzyme released by *P. aeruginosa*. (Chelikani et al., 2004; Mishra and Imlay, 2012).

Figure 3A shows the cyclic voltammogram obtained on a bare pyrolytic graphite electrode bare (OPG) (black line) and modified with CoPc (red and blue lines) in the oxygen-free MH culture medium that was purged with nitrogen for 2 h. The red line corresponds to the cyclic voltammogram obtained when hydrogen peroxide is added in the absence of bacteria. A single peak is observed at -0.64 V, corresponding to the reduction of hydrogen peroxide, as shown in Equation 2. When hydrogen peroxide is added to the MH medium inoculated with bacteria and in the stationary phase of growth, the voltammogram (blue line) reveals a current peak at approximately -0.08 V. This is associated with the reduction of a significant concentration of molecular oxygen (Eq. 1) resulted from the enzymatic activity of catalase (McLeod et al., 1922; Hassett et al., 1997; Baeza et al., 2013; Gulppi et al., 2019). Thus, as previously mentioned, the catalytic activity is assessed by deliberately adding hydrogen peroxide to the culture in the stationary growth phase.

**FIGURE 3:** Potentiodynamic response of OPG bare (black line) and CoPc modified OPG electrode in Mueller Hinton in the absence (red line) and presence (blue line) of *P. aeruginosa* a pH 7.0: **(A)** Cyclic voltammograms recorded at 100 mV/s; **(B)** Square waves voltammograms. Experimental SWV parameters: initial potential -0.2 V, end potential 1.0V, step potential 5 mV, amplitude 20 mV, frequency 25 Hz, equilibration time 5 s.

Further, the square wave voltammetry (SWV) curves in Figure 3B were obtained after adding 30 µL of H_2_O_2_ to the MH culture medium with bacteria under shaking (400 rpm) (blue line) and the bacteria-free broth (red line). In the blue curve, a current peak representing the reduction of oxygen is evident at about -0.08 V, whereas the current peak representing a reduction of hydrogen peroxide to water is smaller than that in the red curve, consistent with the cyclic voltammogram shown in Figure 3A. Comparing Figure 3A with Figure 3B, it is evident that the SWV is much more sensitive for detecting catalase enzyme activity.

Figure 4A shows the voltammograms obtained using a CoPc-modified OPG electrode in a Mueller Hinton medium in the presence of *P. aeruginosa* at different pHs and saturated with oxygen. From the cyclic voltammograms, it is observed that at pH 7.5 (black curve), the first cathodic current peak, which is associated with the reduction of oxygen to hydrogen peroxide, appears at a half-wave potential of 0.18 V, being more positive than those observed at more acidic pHs. On the other hand, from the SWV curves shown in Figure 4B, it is evident that at pH 7.5, the first cathodic current peak appears at more positive potentials (black curve). The behavior described above was very reproducible, suggesting that pH 7.5 favors the electrocatalytic process to reduce oxygen to hydrogen peroxide. At other pH values, the voltammograms are similar, and the differences are mainly in the intensities of the current peaks, the more acidic the environment, the lower the current peaks.

**FIGURE 4:** Potentiodynamic response of CoPc-modified OPG electrodes in Mueller Hinton broth, in the presence of *P. aeruginosa at different pHs*. **(A)** Cyclic voltammograms recorded at 100 mV/s; **(B)** Square waves voltammograms. Experimental SWV parameters: initial potential -0.2 V, end potential 1.0V, step potential 5 mV, amplitude 20 mV, frequency 25 Hz, equilibration time 5 s.

The shift of the first current peak to more positive potentials at ca. 175 mV, and related to the ORR, suggests that catalase activity at pH 7.5 is influenced by the heme group’s orientation and availability. The latter is the active center where hydrogen peroxide is reduced to water according to the oxidative stress described in Equation 3. pH 7.5 seems to be the optimum pH for electron transfer between catalase and hydrogen peroxide. The highest catalase activity at this pH was visibly observed by the abundant generation of oxygen at the electrode surface, which agrees with the O_2_ generation reaction described in Equation 4. Oxygen can be reduced to hydrogen peroxide by reducing O_2_ on the CoPc modified OPG electrode, according to Equation 1. This form of the autocatalytic mechanism was first studied by Busalman *et al.* (Busalmen et al., 2002). Considering this mechanism, the voltammetric response at more acidic pH revealed in Figure 4 is possibly the result of a metal center blocking process, or in other words, of the impediment for hydrogen peroxide to enter the metal center for its reduction to water (Equations 3, 4), which is possibly reflected in a reduction of enzyme (katA) activity (Hassett et al., 1997). This recycling mechanism with O_2_ production promotes oxygen reduction to hydrogen peroxide, which was evident by cyclic voltammetry and square wave voltammetry, CV, and SWV.

### Evaluation of Bacterial Adhesion

#### The Distribution of Bacteria on an Aluminum Alloy Surface

As mentioned in the introduction, one of the primary goals of the present study was to evaluate the influence of pH on the adhesion of *P. aeruginosa* when the microorganism interacts with metal surfaces. This could contribute to understanding the influence of pH on the electrochemical responses presented in Figure 4.

Figure 5 illustrates typical AFM images of bacteria on aluminum alloy surfaces. The roughness of the surfaces is of the order of the bacteria’s thickness, but it can be seen that the cells adapt to the topography of the surface, Figure 5A, exhibiting a soft surface to the external environment. In the case of AA 6063 alloy, Figure 5B, bacteria tend to spread over the flat areas. In Figure 5B, the phase mapping does not present a high contrast between the alloy surface and the bacterial body, indicating that the alloy surface has been covered with some soft components present in the solution or produced by bacteria, which may be associated with biofilm formation.

**FIGURE 5:** Typical AFM images of bacteria adhered to aluminum alloys surfaces obtained in the tapping mode (Left panels: height, amplitude, and phase, respectively. Rightmost panels: three-dimensional profiles of bacteria). **(A)** Set of images at 2 distinct locations of alloy surface AA 2024 inseminated by *P. aeruginosa* bacteria. **(B)** Same for alloy AA 6063. All images were obtained at pH = 7.5.

#### Force, Extension, and Adhesion Energy

Typical force curves are summarized in Figure 6 for both aluminum alloys at pH = 6. First, the averaged force of adhesion is more significant on the AA 6063 surface when compared to that of AA 2024. Second, the extension needed to separate a bacterium from the aluminum surface is also much larger on AA 6063, indicating greater adhesion energy on this surface. In order to gain insight into the difference of adhesion work exhibited by bacteria on the considered aluminum alloy surfaces, the features of force-extension curves are analyzed. Four types of behavior were distinguished. A single jump in the force (Figures 6A,B) indicates a single adhesion point, which was often observed for bacteria interacting with AA2024 alloy surface. The typical force jump was of the order of 0.5 nN. A noticeable feature arising in the bacteria-surface interaction is the extension of filamentary structures whose presence in the force curve is revealed by the typical “worm-like chains” extension (Figure 6C). These structures would extend for about 100 nm and would resist forces before breaking at about 0.5nN. Finally, the pealing mechanism is also exhibited in Figure 6D by the presence of a force “plateau” with the typical amplitude of a fraction of nanoNewton, which takes place over pulling distances of the order of 100 nm. The four types of behavior have nearly equal probability of occurrence.

**FIGURE 6:** Typical force curves obtained at pH 6.0 for AA2024 and AA6063 alloys reveal bacterial adhesion. Single rupture bonds **(A, B)**. Multiple force peaks **(C–G)** forming sawtooth patterns often superimposed onto constant force plateaus **(D)**: as a pilus segment is pulled, a typical nonlinear extension curve characteristic of entropic elasticity **(C–G)** is revealed, while fast unloading signatures the rupture of a pilus bonds at the surface. Zipper-like adhesion reflected by the sequential detachment of multiple pili-surface bonds leading to force plateaus **(D)**, sometimes these plateaus superimpose onto one another **(F–H)**.

Similar features are observed in the interaction of bacteria with AA6063 alloy. The pulling of filamentary structures (Figure 6G) and pealing (Figure 6H) are both detected on this surface. However, the most prominent mechanism responsible for strong adhesion is the interaction of several bacterial elements with the surface (Figures 6E,F). This type of interaction has a strong probability of occurrence at pH close to 6.0. In other words, Figures 6E,F indicate an ensemble of structures supporting adhesion simultaneously; these structures are unlikely focalized adhesion points as those depicted in Figure 6A.

Indeed, for Gram-negative bacteria adhesion is often mediated by a specific interaction between an adhesin, positioned at the distal end of bacterial pilus, and its receptor on the surface of the host tissue (Beaussart et al., 2014). Furthermore, the rod of a pilus contributes with multiple linked sites, which provides additional adhesion to a surface, through specific and unspecific interactions. If the density of points is high the force extension curves reflect a zipper-like adhesion, while a typical entropic elasticity is observed in the low-density case. These features are clearly visible in the force extension curves in Figure 6.

Moreover, the fact that strong adhesion occurs at a given pH, (pH 6) suggests that electrostatic charges on surfaces plays a relevant role regulating cell adhesion.

Alloy 2024 likely provides enhanced negative surface charge, probably due to the absence of copper concerning the AA 6063 alloy. In particular, the layer of aluminum oxide (Al_2_O_3_) generated on these alloys acquires a slightly positive charge at pHs lower than the point of zero charges (ZCP) of the metal oxide, which increases bacterial adhesion. In contrast to what occurs at pHs higher than ZCP (Kosmulski, 2002). In aqueous solutions, the surfaces of materials and bacterial cells are often negatively charged, which causes a repulsive electrostatic force that increases as the surrounding aqueous medium’s ionic strength decreases (van Loosdrecht et al., 1989).

Histograms of adhesion force as a pH function for AA2024 and AA6063 alloy surfaces are summarized in Figure 7. The typical extension of adhesion force is also represented. It is observed that at pH below 6.5, F_adh_, L_adh_, and W_adh_ are higher for AA6063 alloy than AA2024 alloy. The adhesion force (F_adh_) and adhesion length (L_adh_) differ by almost a factor 10, differ significantly, leading to more considerable adhesion differences.

**FIGURE 7:** Histograms for **(A)** adhesion forces, Fadh. **(B)** adhesion work, Wadh, and **(C)** adhesion length, Ladh, for AA2024 and AA6063 aluminum alloy surfaces as function of pH.

The results above can be summarized by presenting the average value over all trials along with the corresponding variance, as indicated through vertical bars in Figure 8. The adhesion work presents a dependence on pH for the surface of AA6063 alloy. A notorious difference in bacterial adhesion between the two aluminum alloys is observed due to variables that influence bacterial adherence and colonization. Specifically, in addition to pH dependence investigated here, the phenomenon and processes of bacterial adhesion should be addressed considering the composition and microstructure of alloys and the microbiological and chemical aspects associated with the cell wall.

**FIGURE 8:** Average work of adhesion for AA2024 and AA6063 aluminum alloy surfaces as a pH function. A clear maximum on the adhesion work is observed for pH near 6.

## Conclusion

• Pyrolytic carbon electrode modified with cobalt phthalocyanine can detect changes in the concentration of hydrogen peroxide associated to catalase activity produced by *P. aeruginosa.*
• The square wave voltammetry technique is more sensitive to detecting the enzymatic activity of catalase than cyclic voltammetry.
• The open circuit potential is sensitive to the cultivation inoculum size. When the inoculum is 1/100 of the culture medium’s total volume, OCP shows the influence of catalase activity.
• The catalase in the MH culture broth at pH 7.5 exhibits a remarkable electrocatalytic activity for ORR compared to that at lower pH values. The availability of the heme group directly affects catalase activity in *P. aeruginosa.*
• The analysis of force curves revealed a pronounced difference in the adhesion of *P. aeruginosa* on aluminum alloys as pH values decrease. A greater adhesion force on the surface of AA-6063 is attributed to the positive surface charge that this alloy exerts on the bacterial cells, reducing the repulsive electrostatic energy barrier to adhere irreversibly to this particular alloy.

## Data Availability

The raw data supporting the conclusions of this article will be made available by the authors, without undue reservation.
